RETRACTED

# B-Ultrasound Image Analysis of Intrauterine Pregnancy Residues after Mid-Term Pregnancy Based on Smart Medical Big Data

**DOI:** 10.1155/2022/9937051

**Published:** 2022-02-16

**Authors:** Huiliao He, Ruixing Liu, Xiuping Zhou, Yinhong Zhang, Beibei Yu, Zhihua Xu, Hu Huang

**Affiliations:** Ultrasound Imaging Department, The Second Affiliated Hospital, Wenzhou Medical University, Wenzhou, China

## Abstract

Abdominal B-ultrasound images of intrauterine pregnancy tissue residues were analyzed to discuss their diagnostic value. With the rapid development of computer technology and medical imaging technology, doctors are also faced with more and more medical image diagnosis tasks, and computer-aided diagnosis systems are especially important in order to reduce the work pressure of doctors. In recent years, deep learning has made rapid development and achieved great breakthroughs in various fields. In medical-aided diagnostic systems, deep learning has greatly improved the diagnostic efficiency, but there are no mature research results for abdominal B-ultrasound image recognition of intrauterine pregnancy tissue residues. Therefore, the study of liver ultrasound image classification based on deep learning has important practical application value. In this paper, we propose to give a CNN model optimization method based on grid search. Compared with the conventional CNN model design, this method saves time and effort by eliminating the need to manually adjust parameters based on experience and has an accuracy of more than 92% in classifying abdominal B-ultrasound images of intrauterine pregnancy tissue residues. The diagnosis of intrauterine pregnancy tissue residues by abdominal B-ultrasound can effectively improve the diagnosis and provide important reference for patients to receive treatment, which has high diagnostic value.

## 1. Introduction

Residual intrauterine pregnancy tissue is a residual appendage or detrusor that remains in the uterine cavity after termination of intrauterine pregnancy, which can cause recurrent vaginal bleeding or uterine infection, and is also an important cause of abortion or postpartum uterine bleeding and infection [1]. Abdominal ultrasound can clearly observe whether there is residual pregnancy tissue in the uterus, and if there is residual tissue, the results of the examination can show the size and location of the residual tissue and its relationship with the myometrial wall of the patient, which can provide accurate and reliable diagnostic basis for medical personnel to formulate appropriate treatment measures and reduce the occurrence of bleeding and infection to a certain extent.

The clinical characteristics of abdominal ultrasound images of intrauterine pregnancy residues after delivery in mid- to late-term pregnancy were studied and the diagnostic effect of ultrasound images was investigated. *Methods.* Forty patients admitted to our hospital with suspected intrauterine pregnancy residues after delivery in mid- to late-term pregnancy underwent ultrasound examination, and those with abnormalities underwent surgical pathological examination. *Results.* The ultrasound images of the 40 patients in this group could be divided into mixed sonographic images (27 cases) and light-dot echo images (l3 cases), of which the conformity rate between mixed sonographic images and pathological diagnosis was 92 stone% (25/27), and the conformity rate between light-dot echo images and pathological diagnosis was 76% (10/13). *Conclusion*. Ultrasound imaging has a good diagnostic effect on the diagnosis of intrauterine pregnancy residues after delivery in mid- to late-term pregnancy and can accurately reflect the specific location, size, and relationship between the residues and the uterine wall while detecting intrauterine pregnancy residues. It is worthy to be widely promoted in clinical practice.

RETRACTED

Intrauterine pregnancy residues are a major cause of postpartum hemorrhage in mid- to late-term pregnancies and are a complication of pregnancy that can lead to serious adverse outcomes. Ultrasound can effectively show whether there are pregnancy residues in the uterus, and if so, the test results can accurately reflect the specific location, size, and relationship with the uterine wall, providing clinicians with a more scientific, accurate, and detailed basis for judgment, thus avoiding the occurrence of bleeding and infection to the greatest extent possible.

In this paper, we improve the method of CNN model design and propose a constraint-based grid search method to design CNN models, which integrates the balance between three different dimensional parameters of CNN models. The CNN obtained after grid search is able to compound and amplify three dimensional parameters by one variable at the same time and then obtain a CNN with the highest accuracy without tedious manual intervention, and the obtained CNN model has higher accuracy and smaller number of parameters compared with the previous chapter.

Compared with the CNN model obtained by tuning the parameters, the experimental method in this paper has four main improvements: (1) the most intuitive is the model accuracy, and the final accuracy obtained in this paper is higher than 92%, and the accuracy is improved. (2) The balance of the three-dimensional variables of CNN depth, width, and input image size can improve the accuracy of CNN classification, and the subsequent experiments also show that the balance will not be destroyed with the CNN scaling. (3) In the experiments of this paper, Flops is introduced in the design of the CNN structure, and the model efficiency is fully considered. (4) The optimal performance of the CNN can be obtained by scaling up the CNN after the grid search, which avoids the complicated and tedious process of tuning the parameters. In order to deeply explore the value of abdominal B-ultrasound in the examination of intrauterine pregnancy tissue residues, this paper performs abdominal B-ultrasound examination on 66 patients with intrauterine pregnancy tissue residues who were included in this study in our hospital between September 2015 and September 2016.

RETRACTED

## 2. Related Work

### 2.1. Current Research Status of Deep Learning in Medical Imaging

Medical imaging technology has made tremendous progress in the past decade or so, but in contrast, the development of computer-aided diagnosis-related technologies has been slightly delayed, especially in medical image analysis. With the development of deep learning in recent years, it has played a significant role in advancing medical image analysis. For example, image segmentation [2], image alignment [3], and image fusion [4] have been used in medical image analysis tasks, and great breakthroughs have been achieved in these tasks.

In the image classification, one of the most common tasks in medical image analysis, supervised learning is mainly used to train the model with annotated training datasets so that the model learns different image features corresponding to different classes of medical images, and after sufficient training, then it classifies unknown test data with high accuracy.

In the task of classifying MRI images of the brain, Akl et al. [5] proposed a deep neural network called multinode network (MSPNet), inspired by the PointNet that can directly process point clouds, which has a high accuracy in identifying Alzheimer's disease and mild cognitive impairment.

For the analysis of breast images, Ji and Kim [6] proposed to use more contextual information for breast image classification, using a convolutional neural network trained on the ICAR2018 dataset to extract tissue features and classify breast cancers into benign, in situ, and invasive breast cancers. In this paper, support vector machines are used to classify the extracted features, but large-scale breast cancer data are lacking. In this paper, the data augmentation technology of illiquid rotating images is used in the training process. Scholten et al. [7] used VGGl6-based convolutional neural network for classification of mammogram images. Garolla et al. proposed a CNN-based CAD technique for breast cancer classification using a pretrained VGG19 network. Mammograms of 69 cancer patients and 27 healthy general individuals were evaluated, and the final sensitivity of the model performance was 0.928 and the specificity was 0991.

RETRACTED

In analyzing images related to ocular region, Grossman et al. [2] used a data-driven approach to classify diabetic retinopathy in color fundus images using a deep learning approach. They trained and tested the model with the public datasets MESSID0R2 and E-ophtha and obtained, respectively. Pratt et al. used a CNN for diagnosing and classifying the severity of diabetic retinopathy in fundus images. Similarly, Barik et al. [8] used the deep CNN structure of ResNet50 to classify fundus images. Scholten et al. [7] proposed a VGG19-based classification system for diabetic retinopathy severity, and they also used 35126 fundus images from the Kaggle dataset for performance evaluation, and their model outperformed traditional methods.

To classify abdominal ultrasound images, Gatford et al. proposed a CNN-based multitask learning framework, in which 187,219 ultrasound images were used in the experiments, and the accuracy of their classification has been higher than that of a professional physician. The deep CNN model used in the article can automatically determine the severity of knee osteoarthritis. In their experiments, a pretrained network trained on ImageNet was used and then fine-tuned on the knee osteoarthritis dataset, and the final CNN model obtained was able to have good classification results. Inspired by the structure of VGG network, the authors used five convolutional layers, ReLU activation function, and 2 *∗* 2 maximum pooling for feature extraction and finally used a long- and short-term memory network with 256 units, and the AUC of the final test result reached 0.83.

### 2.2. Current Status of Research on the Classification of Abdominal B-Ultrasound Images of Intrauterine Pregnancy Tissue Residues

With the maturation of medical imaging technology, ultrasound has become the most common modality to examine fatty liver. The algorithm adopts manual extraction of the attenuation coefficient of the image and uses a mathematical statistical framework to detect fatty liver. Qayyum et al. proposed a “grayscale correlation grade” through regions of interest in multiple ultrasound images to indicate different fatty liver classes. Mihailescu et al. calculated the attenuation values from regions of interest and used a mathematical statistical framework to detect fatty liver. “Mihailescu et al. calculated attenuation values from regions of interest and used random forest to classify ultrasound images of intrauterine pregnancy. Vicas et al. used attenuation coefficients, fitting errors, etc., as feature sets and used SVM classifier to perform quantitative analysis of fatty liver. The principle of quantitative analysis used in this paper is to extract several features of ultrasound images in the gray-scale covariance matrix such as autocorrelation and signal-to-noise ratio and using logistic regression to determine the severity of fatty liver. The scatter coefficient of abdominal B-ultrasound images of intrauterine pregnancy tissue remnants can also be used to quantify the fat content of the liver.

RETRACTED

In all of the above methods, features of ultrasound images need to be extracted manually before performing classification experiments. CNNs have surpassed many traditional algorithms in the current field of computer vision tasks. Therefore, for ultrasound in utero pregnancy ultrasound image classification, CNN can be considered for the classification task. CNN does not require complex and tedious feature extraction process like the traditional methods in the previous literature and can learn texture features directly by convolutional operations and then perform classification, but currently CNN-based recognition methods have not been fully applied to ultrasound in utero pregnancy ultrasound images.

## 3. Optimization Method of CNN Model Based on Grid Search

### 3.1. Determination of Baseline CNN Model

The scaling of the CNN model does not change the specific computational operations such as convolution, pooling, or normalization in the CNN but mainly changes the depth and width of the model and the size of the fatty liver image size. Therefore, it is crucial to have a fully trained baseline CNN network, which is the basis for the later CNN model scaling and directly related to the performance of the CNN model after scaling.

### 3.2. Optimization of CNN Models Based on Grid Search

However, some current studies have shown that there is often a certain coupling relationship between the width and depth of CNN models *m*, and the increase of its accuracy may be limited by adjusting a single parameter of the model, so it is important to balance different dimensional parameters of CNN to improve the efficiency of CNN.

Optimization of the CNN model using a grid search-based approach starts with determining a well-trained CNN baseline model. Then, a grid search is performed to determine an optimal CNN given the maximum number of parameters, and a formula is proposed to balance the relationship between the parameters of each dimension of the CNN during the search process. Finally, the searched CNN model is scaled up and the accuracy is improved.

RETRACTED

In Figure 1, the first step first compares the scaling of the parameters in a single dimension with the composite scaling to verify the proposed conjecture of the existence of a coupling relationship between the parameters. The second step determines the optimization objective of the CNN model. In the third step, given the computational resources, a small-scale search is performed to determine a scalable network model under the constraint of a formula that balances the parameters of each dimension of the CNN. Finally, the model determined by the grid search method is scaled.

#### 3.2.1. Composite and Single Scaling of CNN Parameters in Different Dimensions

The design process of CNN models needs to pay attention to the computational resources required for training, because in the actual application process, many embedded devices often have limited computational power. Lightweight network models are also becoming a hot topic of research. Some lightweight networks are more accurate than structures with a large number of parameters, but require less computational power, and these network models are more practical in practical engineering applications.

In this experiment, image size is added as a factor to explore the relationship between the three dimensions of network width, depth, and the size of the input image. Empirically, the larger the image size is, the more layers it may need to increase the perceptual field of the model, and also the larger the width to capture more detailed feature information on the image. In the process of deep learning research, many CNN models with very large number of parameters have emerged. Although they can achieve very good models, they cannot provide large enough computational resources to meet the requirements in practical application scenarios and usually reduce the number of parameters of the model at the expense of accuracy through methods such as model compression.

At present, the criterion used more often in research to evaluate the arithmetic power required for CNN models is Flops. The complexity of a model can also be judged by Flops, and for a certain convolutional layer of CNN, it is calculated as shown in the following equation:

(1) $$\begin{array}{c} \text{Flops}=H{\;}^{*}W{\;}^{*}n{\;}^{*}\left(h{\;}^{*}w{\;}^{*}c+1\right). \end{array}$$

There are various methods of model scaling; ResNet models can be scaled down to ResNet-18 or scaled up to ResNet-200; WideResNet and MobileNet can scale the model by width. The width and depth of the CNN model play a very important role in the expressiveness of the CNN model, as demonstrated in the experiments in the previous section. However, the model for classifying abdominal B-ultrasound images of intrauterine pregnancy tissue residues needs to be further investigated to obtain better efficiency and accuracy of the CNN model.

RETRACTED

Instead of scaling the model width or number of layers singularly by the control variables method, the experiments in this section use a composite scaling method to simultaneously scale the width and depth parameters and then observe the changes in model performance while adding the input image size as a factor. In Figure 2, a baseline network and the composite scaling of the model parameters based on it are presented, and in Figure 3, the scaling methods of the model width, depth, and image input size are depicted in detail, respectively.

In Figure 2, the composite scaling is mainly to change the width, depth, and input image size of the CNN model structure simultaneously. In the study of the previous section, the model optimization of CNN is all based on manual experience of scaling in the direction of a single dimension. In this section, it is experimentally demonstrated that changing the parameter sizes of different dimensions of CNN simultaneously is more effective than changing the parameters of a single dimension for improving the accuracy of CNN models.

Figure 3 shows schematic diagrams of single dimensional scaling of the CNN model structure using different widths of the network structure, depth, and size of the input image size for training, respectively. The depth of the network model is one of the main factors that affect the performance of the main CNN model.

Figure 4 is scaling based on the depth (d) of the baseline CNN model. In Figure 5, the curves represent the effect of model width *w* on accuracy, which is the same as model depth d, same as different model widths obtained by multiplying *w* with different coefficients with the width of the baseline model. As the width *w* increases, Flops keeps increasing and the accuracy rate keeps rising, but the accuracy rate will gradually level off. The experiments for the size of the input image are shown in Figure 6. There are four different sizes of images, 20 *∗* 20, 28 *∗* 28, 35 *∗* 35, and 40 *∗* 40, and the Flops increase as the size of the image size increases. When the image size is 20 *∗* 20, the accuracy rate is significantly lower compared with the accuracy rate of other experimental results, and the accuracy rate of the other three types of image sizes is basically the same with no significant changes.

However, the accuracy improvement of this type of method is relatively limited, and the accuracy rate tends to stabilize after rising to a certain value, and then parameter adjustment to increase Flops does not improve the accuracy rate significantly. Therefore, these methods have some limitations.

RETRACTED

Single dimensional scaling can improve the accuracy of CNN models, but there are shortcomings and the improvement of model accuracy tends to flatten out. In this section, compound tuning of model parameters is used to explore whether there is a coupling relationship between different parameters and whether it is more effective than single dimensional tuning for CNN models to improve the accuracy of identifying ultrasound images of intrauterine pregnancy. Some studies have mentioned the relationship between depth and width of CNN models and have also tried to balance the width and depth of CNNs, but all of them require a lot of tuning based on manual experience. There is a certain coupling between different dimensions of CNNs such as width and depth. For images with higher resolution, a deeper network may be needed to extract deeper features, while a wider network may be needed to extract more different features.

The above is based on the experience of tuning the parameters of the CNN model, and the simultaneous tuning of different dimensional parameters requires coordination and balance. To verify whether the CNN model for ultrasound image recognition of intrauterine pregnancy conforms to this basic hypothetical conjecture, the following experiments were conducted. The specific experimental results are shown in Figure 7, using two variables to simultaneously vary the depth of the CNN model with the size of the input image.

In Figure 7, four sets of different combinations of parameters are used to experiment on the baseline CNN model, which verifies the preliminary conjecture of the previous one. The composite scaling has a certain effect on the accuracy improvement related to the highest accuracy rate of more than 88%, and the highest accuracy rate of the previous experiment is only 86%. The variables, depth, which represent the depth of the CNN model are 0.5 and 1.25 to scale down and scale up the original baseline CNN model, respectively. Two different sizes of image 28 *∗* 28 and 35 *∗* 35 are used here. By combining the variables, and then conducting experiments to obtain the abovementioned graph of the relationship between Flops and accuracy, the accuracy rate is also gradually increasing with the increase of the computational volume, and the final accuracy rate is higher than that of the single dimensional scaling effect.

#### 3.2.2. CNN Optimization Objective Based on Grid Search

The main consideration of grid search CNNs is the balance relationship between the size of Flops and parameters. The goal of the grid search is to find the scalable CNN with the highest accuracy under the balance condition as well as the fixed Flops constraint.

RETRACTED

The first is to clarify the CNN optimization objective combined with the computational volume Flops; for the CNN convolutional layer, assume a convolutional layer operation formula as *Y*_*i*_= *F*_1_(*X*_1_), where *i* represents the *i*-th layer convolution, *x*_1_ represents the input of the *i*-th layer convolution, and *K* represents the convolutional layer output. The whole CNN model operation can be regarded as

(2) $$\begin{array}{c} N=F_{k}\left(X_{k}\right)*F_{k-1}\left(X_{k-1}\right)*\ldots *\;F_{1}\left(X_{1}\right). \end{array}$$

In the actual CNN model framework, there will be many convolutional layers, which basically share the same type of convolutional operations, so the whole CNN model can be reduced to the following formula:

(3) $$\begin{array}{c} N=\prod_{i}F_{i}\left(X_{\left(h_{i},w_{i}\cdot c_{i}\right)}\right), \end{array}$$

in which *h*_*i*_ and *w*_*i*_ represent the size of the convolution kernel of the *i-*th convolution layer, and *c*_*j*_ represents the number of convolution kernels, i.e., the width of the *i*-th layer. Unlike the previous CNN model structure design, this part does not change the convolutional computation part *F*_1_ but focuses on changing the model depth, width, or resolution size of the image and does not change the specific convolutional computation for.

Here, for CNN model optimization under resource constraints, the main aspects include the following: (1) maximizing the CNN model accuracy, which can be expressed as the following equations:

(4) $$\begin{array}{c} \max\;\mathrm{Accuracy}\left(N\left(d,w,r\right)\right), \end{array}$$

(5) $$\begin{array}{c} N\left(d,w,r\right)=\prod_{i}F_{i}\left(X_{\left(d\cdot h_{i},w\cdot w_{i},r\cdot c_{i}\right)}\right). \end{array}$$

The constraints are mainly Flops and number of parameters. The CNN model searches for the optimal network structure under the constraints of certain Flops and model parameter size as shown in the following equations:

(6) $$\begin{array}{c} \text{Memory}\left(N\right)<{\text{target}}_{\text{Memory}}, \end{array}$$

(7) $$\begin{array}{c} \text{Flops}\left(N\right)<{\text{target}}_{F}\text{lops.} \end{array}$$

In theory, the larger the number of CNN model parameters, the greater the computational power required for training, and the higher the accuracy rate will be gradually. The goal of the summary formula optimization is to traverse the search to the CNN model structure with the highest accuracy rate for classifying ultrasound images of intrauterine pregnancy under a fixed Flops constraint. CNN needs to fully take into account the Flops constraint, which mainly serves to narrow the parameter space in the grid search and determine the scalable CNN network model more quickly.

RETRACTED

## 4. Experimental Results and Analysis

### 4.1. Comparison of CNN Optimization before and after

Firstly, in order to verify the effectiveness of the model scaling method in this experiment, a comparison of the accuracy of the scaling method in this experiment with that of the scaling performed in a single dimension was first performed under the same Flops required for CNN. The three methods are increasing only the depth of CNN, i.e., the number of layers, increasing only the width of CNN model, and the method proposed in this experiment, compounding three dimensional parameters to expand the CNN model at the same time.

As can be seen from the experimental results in Table 1, compared to the baseline model, the single dimensional scaling brings an improvement in accuracy and requires more computational resources. However, with almost equal Flops, the composite scaling approach in this experiment is again able to be significantly better than the single dimensional results, with an accuracy improvement of about 3 percentage points. The CNN model structure designed by the experimental method is more effective and can obtain higher accuracy at the same Flops.

Figure 8 shows the visualization results of the different methods, from which it can be seen that the composite scaling method proposed in this paper can more effectively capture the finer textural features of the abdominal B-ultrasound images of intrauterine pregnancy tissue residues.

### 4.2. Composite Amplification Experiment of CNN Model

By the previous method of grid search, the values of the three parameters are determined based on the baseline CNN model *α*=1.5, *β*=1.71, and *γ*=1.25, and these three variable values correspond to a specific CNN structure.

The variable values of each dimension are obtained, and there will be decimal values in the calculation process, but the actual variable values should not be decimal values. At this time, the treatment is that the decimal values are rounded up and down, and then the accuracy of the two parameters corresponding to the CNN model is compared separately, and then it is determined which integer is taken. In Figure 9, for the scaled-up CNN model, the names of the models in this experiment are directly presented as numerical numbers, and the values of the three variables are the final rounded results.  Table 2 shows the specific parameters of the magnified series model.

In total, five scaling-ups were done for the grid-searched CNNs, because in the actual experiments, it was found that the accuracy growth of the models tended to level off and basically did not continue to increase when the scaling-up factor continued to increase. The Hops of the CNN models gradually increased, and the Flops of different CNN models were distributed in different intervals of the horizontal coordinates of Figure 9. The scaling up of the optimal CNN model searched by the grid only increases the three dimensional variables of depth, width, and size of the input intrauterine pregnancy ultrasound image, and the other parameters of the remaining CNNs remain unchanged. The specific classification accuracy of this series of CNN models is shown in Figure 9, which gives the specific trends of the Flops of the CNN models and the corresponding classification accuracy. Figure 9 shows the model Flops and accuracy after scaling up by the scaling factor, and it can be seen by the line graph that after scaling up the model by the scaling factor, the accuracy grows with the growth of Flops, and the highest accuracy of the final CNN model is over 92%.

RETRACTED

In this paper, the proposed method based on grid search, which balances the parameters of each dimension of CNN, is more efficient and the accuracy of the model is higher with the same number of parameters.

## 5. Case Study

### 5.1. Clinical Information

In this study, the clinical data of 40 postpartum patients with mid- to late-term pregnancy who came to our hospital from January 2014 to January 2015 were retrospectively analyzed. The age of the patients ranged from 22 to 41 years. The main postpartum symptoms included continuous or indirect vaginal bleeding, lower abdominal pain, amenorrhea, and elevated body temperature. In addition, 27 patients had irregular vaginal bleeding or amenorrhea, and 13 patients had lower abdominal pain and fever. The patients were routinely examined by transabdominal pelvic ultrasound. In the absence of vaginal bleeding and obvious signs of infection, transvaginal ultrasound can be combined with the examination.

It is necessary to drink a lot of water before the examination. Only when the bladder is filled to a certain level can the uterus be squeezed from deep in the pelvis to the lower abdomen and the uterine cavity be observed with ultrasound. A combined supra-abdominal scan of the uterine adnexa was performed via the abdominal wall at the pubic bone, focusing on the changes in the uterine cavity and the endometrial echoes.

This method does not require holding urine, and because it is close to the uterus and ovaries, the images are clear and have high resolution, making the results more accurate. However, it is not suitable for people with vaginal bleeding, such as menstrual periods or irregular vaginal bleeding. It is also not suitable for people with infectious diseases, such as vaginitis and sexually transmitted diseases. It should also be used with caution in cases of other cervical, vaginal, and vulvar diseases to prevent infection and bleeding.

RETRACTED

### 5.2. Results

In the present group of 40 patients, ultrasound images showed mixed acoustic images (27 cases) and echogenic images of light clusters (13 cases), with a diagnostic compliance rate of 926% (25/27) and 76.9% (10/13). 40 cases showed an enlarged uterus with normal uterine morphology, indistinct endometrial lines, and homogeneous echogenicity of the myometrial wall. 40 cases showed inhomogeneous high, medium, and low echogenic light clusters in the uterine cavity. In 34 cases, the morphology was irregular, accounting for 80% of the cases, and the size was between 1 and 4 cm. All clusters were of varying echogenicity and irregular borders; in 6 cases, strong echogenicity was seen with acoustic shadowing. The residues were confirmed to be embryonic tissues and old blood clots, ranging from 20 to 2259 in volume, and the pathological examination was performed on degenerated necrotic meconium, and in 8 cases, there were fetal bones in the residues. After the treatment of uterine evacuation, 25 of the 40 cases had their vaginal bleeding stopped and pain relieved after 1 time evacuation; 12 cases had 2 times evacuation and 3 cases had 3 times evacuation until the uterine size returned to normal and there was no abnormal strong echo in the uterine cavity.

## 6. Discussion

The intrauterine pregnancy residues are a common cause of postabortion and late postpartum uterine bleeding or infection. The analysis showed that patients with mixed echogenic ultrasound diagnostic images had a higher diagnostic compliance rate because they had more residues in the uterine cavity, which provided a reliable basis for the treatment of uterine evacuation and also effectively prevented intrauterine infection. For patients with ultrasound diagnostic images of light cluster echogenicity, which is difficult to distinguish from blood clots, the compliance rate is reduced. For such patients, treatment with contraction agents and anti-inflammatory drugs can be performed first, and then curettage can be performed after failure, which avoids unnecessary trauma to the uterine cavity and minimizes the patient's pain.

In summary, ultrasound testing can provide a more scientific and reliable clinical basis for accurate diagnosis of intrauterine pregnancy residues after delivery in mid- to late-term pregnancies and can also perform ultrasound-guided uterine evacuation for patients, effectively avoiding the blindness of previous surgery, improving the success rate of surgery, and reducing the occurrence of various complications, which is worthy of wide clinical use.

RETRACTED

## 7. Conclusions

Intrauterine pregnancy residue is a dangerous disease in obstetrics and gynecology, mainly caused by excessive curvature of the uterus. It is commonly seen in patients who have had a medication abortion at a long gestational age, in those who have undergone a poorly performed abortion, in those who have undergone an induction of labor in mid-pregnancy, resulting in adhesions between the fetal membranes and the placenta, and in those who have had abnormal changes in the morphology of the uterine cavity. Patients are prone to recurrent vaginal bleeding after the onset of the disease, which has a significant negative impact on the patient's health, so it is important to diagnose the patient promptly and accurately

The internal echogenicity is rougher. In addition, in patients with small pregnancy residues, one or more small substantive plaques can be observed in the mucosal layer of the uterine cavity. If the patient has a residual pregnancy tissue in the uterus along with fluid in the uterine cavity, the residue may be visualized as a ring, strip, or irregularly separated fluid-free area between the residue and the contralateral uterine wall, and the residue may appear as a pike, strip, mass, or peninsula or be flattened, with an echogenic image hyperechoic.

It can be seen that the diagnosis of intrauterine pregnancy tissue residues by abdominal B-ultrasound can effectively improve the diagnostic results and provide important reference for the later treatment of patients, which has high diagnostic value.

Abdominal B-ultrasound images of intrauterine pregnancy tissue residues were analyzed to explore their diagnostic value. With the rapid development of computer technology and medical imaging technology, doctors are also faced with more and more medical image diagnosis tasks, and computer-aided diagnosis systems are especially important in order to reduce the work pressure of doctors. In this paper, we propose to give a CNN model optimization method based on grid search. The method first determines a baseline CNN model and then optimizes it by approximate Flops per second, and for intrauterine, the accuracy of abdominal B-ultrasound image classification of pregnancy tissue remnants was over 92%. The diagnosis of intrauterine pregnancy tissue residues by abdominal B-ultrasound can effectively improve the diagnosis and provide important reference for patients to receive treatment, which has high diagnostic value.

## Figures and Tables

**Figure 1:** Main model.

**Figure 2:** Model scaling; (a) baseline model; (b) composite scaling based on baseline model.

RETRACTED

**Figure 3:** CNN model structure optimization methods in different dimensions; (a) model width scaling; (b) model depth scaling; (c) input image size scaling.

**Figure 4:** Scaling based on the depth (d) of the baseline CNN model.

**Figure 5:** Scaling based on the width (w) of the baseline CNN model.

**Figure 6:** Different image (R) sizes based on the input of the baseline CNN model.

**Figure 7:** Composite scaling based on baseline CNN model with different scaling parameters.

**Figure 8:** Visualization of abdominal B-ultrasound images with composite scaling of other methods.

**Figure 9:** Amplification factor vs. Flops and accuracy line graph.

**Table 1:** Classification results of different methods.

CNN model	Flops (million)	Accuracy (%)
Baseline CNN model	2.4	85.9
Only expand the depth of CNN	18.2	87.6
Only expand the width of CNN	18.3	87.3
Compound amplification	17.9	90.5

**Table 2:** Specific parameters of the scaled-up series of models.

Model	Amplification factor (*θ*)	Depth (d)	Width (W)	Image size (c)	Flops (million)
CNN01	1.5	4	81	28 *∗* 28	4.7
CNN02	2	4	108	35 *∗* 35	6.8
CNN03	2.3	5	124	35 *∗* 5	14.6
CNN04	3.7	6	200	40 *∗* 40	17.8
CNN05	4.1	6	221	40 *∗* 40	24.9

## Data Availability

The simulation experiment data used to support the findings of this study are available from the corresponding author upon request.
